The article "A Preliminary Study on the Dramatic Factors of Ancient Chinese Poetry under the Changing Geographical Environment" was retracted in 2023. Reasons: signs of a paper mill; suspected computer-generated content; unreliable results or conclusions; concerns about the data.

# A Preliminary Study on the Dramatic Factors of Ancient Chinese Poetry under the Changing Geographical Environment

**DOI:** 10.1155/2022/4220059

**Published:** 2022-07-30

**Authors:** Yanfang Liu

**Affiliations:** School of Communication, Shanxi Normal University, Taiyuan 030031, China

## Abstract

The formation of Chinese traditional culture is influenced by many factors, and the natural geographical environment is an important factor. Because a country's status is based on its geographical environment, it affects many aspects, such as economic composition and national psychology. As one of the expression forms of traditional Chinese culture, ancient Chinese poetry has a great influence on the emergence and development of Chinese traditional culture. Therefore, this paper mainly discusses the specific influencing factors of the drama of the ancient Chinese poetry, and the preliminary study of it is of certain significance to the development of Chinese traditional culture.

## 1. Introduction

The genre of quatrains was finalized in the Tang Dynasty and developed almost to perfection [1]. Tang Dynasty poets not only used quatrains to describe scenery and objects but also overcame the limitation of short quatrains and used superb artistic generalization to write people in quatrains [2]. Some masterpieces can even display situations, plots, and scenes similar to drama literature in a limited space discourse [3]. It can be said that there are not only “paintings” in poems and “people” in poems but also “plays” in poems. Various literary styles always influence and penetrate each other [4]. Quatrains have been recited in the population for a long time, and they are appreciated by both the refined and the popular [5]. Discussing their dramatic factors has a certain significance for the initial study of the dramatic factors of ancient Chinese poetry under the changing geographical environment and deserves due attention.

A nation forms a stable national culture, and its influencing factors are multifaceted which include political system, economic foundation, and natural environment. Among them, the natural geographical environment occupies an important position [6] because the place where a nation stands is based on its geographical environment and it affects many aspects such as economic composition and ethnic psychology [7]. The reason why Chinese traditional culture can be maintained for a long time is that it will not be interrupted like other ancient civilizations and it has formed a Chinese culture dominated by farming culture, a small-scale peasant economy that is economically self-sufficient, and a conservative and closed national psychology. The natural geographical environment is inseparable [8].

The article "A Preliminary Study on the Dramatic Factors of Ancient Chinese Poetry under the Changing Geographical Environment" was retracted in 2023. Reasons: signs of a paper mill; suspected computer-generated content; unreliable results or conclusions; concerns about the data.

In terms of geographical environment, the scope of the traditional Chinese regime is relatively fixed. The main scope is roughly the west of the Pacific Ocean, east of the Qinghai-Tibet Plateau, north of the South China Sea, and south of the Mongolian Plateau, which is the “Huaxia” in history, which also constitutes China [9]. Among them, the most stable ruling area is south of the Yinshan Mountains and the middle reaches of the Liaohe River and the Qinghai-Tibet Plateau and the east of the Hengduan Mountains in the mainland of China [10]. It is concentrated in the middle and lower reaches of the Yellow River and the middle and lower reaches of the Yangtze River [11]. This part of the territory also constituted the original cradle of the Chinese nation. It can be seen that this part of the region is mainly located in the northern temperate zone. This part of the region has a warm climate and fertile soil, ideal for agricultural development [12]. Located in the interior of the Eurasian continent, the area is closed, less subject to external intrusion, and cultural traditions can be continued. It has had a significant impact on the emergence and development of Chinese traditional culture [13]. As an indispensable part of Chinese traditional culture, ancient poetry and its natural geographical environment also have a profound influence on its development and cultural evolution.

## 2. Natural Geographical Environment

Under different natural and geographical environments, the forms of folk songs are also different, as shown in Figure 1.

### 2.1. The Influence of Natural Geographical Environment on the Formation of Chinese Poetry

Throughout the development history of human civilization and culture, we can see in Figure 2 that those great civilizations in ancient times were mostly concentrated in the river basin, which is called “the river civilization.”

In ancient China, the topography of the middle and lower reaches of the Yellow River and the middle and lower reaches of the Yangtze River was flat and dominated by plains. The climate dominated by the north temperate zone is warm and humid, with abundant water sources and rain and heat in the same season [14]. At that time, the Loess Plateau was still a forest. Under such unique conditions, agriculture developed rapidly and it became the initial cradle of Chinese civilization [15]. Many modern archaeological documents and archaeological discoveries have confirmed that the central areas of ancient civilizations such as Xia, Shang, and Zhou were the central and northern parts of today's Henan Province, southern Shanxi Province, the Guanzhong Basin in Shaanxi Province, the southwestern part of Hebei Province, and the western part of Shandong Province. It was also the region with the most favorable natural environment at that time. Ancient Chinese ancestors lived and multiplied on this land [16]. The soil blown from the western plateau allows the nutrients of the land here to be replenished every year, instead of abandoning and looking for other land every year, the sustainable development of agriculture is guaranteed, agriculture is developed, and various farming tools appear very early [17]. Then, it is not surprising that advanced farming civilization appeared in the Central Plains. The economic, demographic, and geographic foundations for the emergence of Chinese culture are already in place. Since then, China's ancestors have worked on this land for generations, forming the initial prototype of Chinese civilization. Before the emergence of industrial civilization, we observe that which country is the most developed agricultural economy and which country is the most powerful. With the support of China's geographical location, China's agricultural civilization has always been very developed, and it has always occupied a far leading position in the world [18].

The article "A Preliminary Study on the Dramatic Factors of Ancient Chinese Poetry under the Changing Geographical Environment" was retracted in 2023. Reasons: signs of a paper mill; suspected computer-generated content; unreliable results or conclusions; concerns about the data.

Natural ecology is inextricably linked with ancient Chinese poetry. Ecological environment is the basic place on which human beings survive and develop, and it also provides the best opportunity for ancient poets' literary creation and an important content of literary performance. A large number of various natural scenery, animal, and plant images into poetry make ancient poetry present “green,” vibrant characteristics, for readers to show a colorful ecological picture scroll. At the same time, the poetry creation of ancient poets makes the ecological things that originally belong to nature into people's aesthetic cultural vision, thus attaching a strong human culture and poetic color.”

### 2.2. The Natural Geographical Environment Enables the Development and Continuation of Chinese Poetry

With the development of agriculture, the Chinese nation can no longer be satisfied with the land in the Central Plains. Therefore, in the ancient poetry at this time, the characteristics of various nationalities and different geographical environments began to appear [19]. Although the development speed is relatively slow, Chinese poetry has been developing forward with the support of agricultural economy. From the perspective of surrounding and external, China's geographical environment has effectively guaranteed the continuation of Chinese poetry [20]. To the east of the territory is the Pacific Ocean, to the south is the South China Sea, and to the west is the Qinghai-Tibet Plateau. This will completely surround China. The barrier of the natural geographical environment makes this area rarely invaded by foreigners, which provides an external guarantee for the development of culture. At this time, only the north had no security and it was exposed to the nomads in the north, which posed a great threat to the survival of the entire civilization. This is indeed the case in history. In the case of underdeveloped transportation in ancient times, various powerful empires in the distance could not quickly reach China and conduct wars. Most of the harassment suffered in China's history came from the north. The rulers of China thought of a way to build the Great Wall. In this way, China's four conveniences have barriers. Such a historical background and geographical environment characteristics also promote the prosperity of contemporary poetry.

The article "A Preliminary Study on the Dramatic Factors of Ancient Chinese Poetry under the Changing Geographical Environment" was retracted in 2023. Reasons: signs of a paper mill; suspected computer-generated content; unreliable results or conclusions; concerns about the data.

Ancient Chinese poetry is inextricably linked with the natural ecology. The vibrant and colorful ecological world is the best opportunity to inspire the poetry of ancient poets and constitutes an important content of their literary expression. Various kinds of mountains, rivers, natural landscapes, and animal and plant emotions have entered the poet's pen and become a series of colorful poetic images. Ancient poems are “green” because of these natural images, showing readers a colorful ecological picture scroll. At the same time, natural images also enter people's aesthetic cultural vision because of the poet's attention and aria, thus attaching the color of human culture, poetic, and even personification in addition to their own natural attributes. In the ancient Chinese aesthetic culture tradition, some natural objects such as plum and bamboo carry the profound psychological accumulation and rich humanistic emotion connotation of the Chinese nation. The marriage between ancient poetry and natural ecology makes them complement each other.

### 2.3. The Natural Environment Has Created the Diversity of Chinese Poetry

The vastness of China's territory has been maintained, which is also rare in the history of the world. Such a vast territory has extremely diverse topography, including mountains, rivers, plains, and plateaus. Traffic in ancient times was inconvenient, and such terrain was likely to create an insurmountable barrier. There is a lack of communication between various cultural areas, and the differences are becoming larger and larger, resulting in the formation of cultural styles with different characteristics, as shown in Table 1.

Another example is that due to the barrier of the Hengduan Mountains, the transportation between ancient Sichuan and the Central Plains was very inconvenient, so it was called “natural danger.” Judging from the Sanxingdui cultural relics excavated by archaeology, the bronze ware technology in the ancient Sichuan Basin was extremely developed and the stratum system was also different from that in the Central Plains. In Lingnan, further south, the difference is even greater. Due to the proximity to the ocean, frequent exchanges with the outside world, and the difficulty of reaching the control of the Central Plains dynasty, the culture here is relatively open and people's concepts are also very different from the Central Plains tradition. It is not surprising that China's early foreign trade and opening of ports occurred in Guangdong Province. It is this diverse natural and geographical environment that has created such different cultures of various ethnic groups and regions, which makes Chinese poetry present a splendid feature. The degree of cultural diversity is also amazing in the world.

The article "A Preliminary Study on the Dramatic Factors of Ancient Chinese Poetry under the Changing Geographical Environment" was retracted in 2023. Reasons: signs of a paper mill; suspected computer-generated content; unreliable results or conclusions; concerns about the data.

Ancient natural environment beautiful, diverse ecological conditions constitute a good background of the poet creation, poets capture all kinds of natural poetry, and poetry language is no longer just an abstract symbol, we can see the colorful ecological world and vivid harmony between man and nature. The rich and colorful green ecological factors in nature enter people's poetry, making the poetry “green,” and the picture presented by the poetry becomes more gorgeous and colorful.

### 2.4. The Natural Environment Has Had a Significant Impact on Chinese Politics and National Psychology

Such a geographical environment has played a certain role in blocking external aggression, but it has also resulted in the superstability and isolation of Chinese politics and the arrogance and conservativeness of national psychology. If there is no crisis caused by external invasion, a dynasty can basically continue relatively smoothly. Changes of dynasty are infrequent. Moreover, the political system will not change much. Political stability creates cultural stability. The mainstream of China's feudal culture for more than two thousand years is Confucian culture, which lacks changes. They were proud of their abundance of products and considered themselves “the kingdom of heaven,” which resulted in political stagnation and lack of progress. It is reflected in the national psychology that this safe environment makes the people comfortable with the status quo and cling to the farming economy. In traditional Chinese concepts, family, clan, and blood ties are particularly valued, and they are inseparable from the development of farming and economic development caused by the natural environment. “Relocating in a peaceful land” and “not traveling far away” are very important psychological concepts of traditional Chinese people. Unlike the western marine culture, which is full of changes and adventures, because of the superior natural environment, China has always been in a state of self-sufficiency, and the rulers and people are satisfied with the status quo. While the agricultural economy is stable, it also results in a conservative and autistic national psychology. In this context, contemporary poetry can also reflect the ethnic psychology of that time. For example, caused by the present natural scenery homesickness, pregnant, hurt yourself, or with the help of the natural scenery to abstract, difficult to directly say ideas in the long-term poetry creation practice gradually become a poetry generation mode, and many natural objects also gradually attached to the specific cultural psychological connotation and from generation to generation continue. We can pick up an ancient poem and almost always find some natural images. These images come from the natural ecological world, but also have a certain cultural significance.

The article "A Preliminary Study on the Dramatic Factors of Ancient Chinese Poetry under the Changing Geographical Environment" was retracted in 2023. Reasons: signs of a paper mill; suspected computer-generated content; unreliable results or conclusions; concerns about the data.

## 3. Dramatic Factors in Tang Dynasty Quatrains

The heyday of poetry was in the Tang Dynasty in China, which was mainly influenced by the historical background and natural environment at that time, which made all the ancient poems of the Tang Dynasty show very dramatic characteristics. The dramatic factors in the poems of the Tang Dynasty are shown in Figure 3.

### 3.1. Dramatic Scenes in Tang Dynasty Quatrains

Due to the limitation of space, the quatrains of the Tang Dynasty often write lyrical emotions in concentrated scenes, so a situation similar to a drama often occurs: time, place, characters, events, and conflicts are very concentrated and reflected in the form of an instant. This dramatic situation is not only an opportunity for the outbreak of dramatic conflicts but also an objective condition for the characters to produce unique actions. In fact, in the quatrains of the Tang Dynasty, most of the characters that are prompted by this dramatic situation are “still actions” similar to the dramas, so what we see in the quatrains of the Tang Dynasty are mostly dramas similar to the “silence” or “pause” in the dramas situation. Readers can also see the same situation in ancient Chinese drama literature.

The characteristics of dramatic situational concentration in the quatrains of the Tang Dynasty are very prominent. Good quatrain writers are particularly good at capturing moments to construct dramatic situations. Just as Ye Weilian said, “A lyric (lyric poem) often captures a moment of time that contains rich content,” this moment contains events that imply the development of many lines before this moment, and there are many linear events that may develop at this moment. First, Tang Chinese quatrains often use moments to construct dramatic situations. In this particular moment, time, place, people, events, and conflicts are very concentrated.  Table 2 lists where the dramatic scenes of Tang Dynasty poetry generally appear.

The article "A Preliminary Study on the Dramatic Factors of Ancient Chinese Poetry under the Changing Geographical Environment" was retracted in 2023. Reasons: signs of a paper mill; suspected computer-generated content; unreliable results or conclusions; concerns about the data.

Compared with ordinary life situations, the biggest difference between dramatic situations is that it is an opportunity for the outbreak of dramatic conflicts, for example, Wang Changling's “The Resentment of the Bodhisattva”: “the young woman in the boudoir does not know her sorrows and she puts on makeup in the spring. She suddenly sees the color of willows on the street and regrets teaching her husband and son-in-law to find a marquis. “Cuilou” and “Spring Day” by Yangliuqingqing on the street: the inner conflict between the young woman in her boudoir and the young woman's desire to “want her husband to find a lord” and her longing, who went upstairs alone, constitute a concentrated dramatic situation. Before this spring day, the young woman's thoughts were dominated by her “want her husband to find a title.” Hou's heart, so at the beginning of the poem, she shows “no worries,” even if she is alone, she “makes up on the green building” to appreciate the beautiful spring. But in a specific situation—“the color of willows on the street” “Inspired, she may have thought of the beauty and ephemeral nature of youth and spring, and the beauty of youth and spring that no one can appreciate …. so, the longing that had been lurking in her heart surfaced, and it was associated with fame and fortune.” There is a strong conflict in the heart: “repent and teach the husband and son-in-law to find a lord,” the specific situation finally prompted the outbreak of the dramatic conflict. Most of the dramatic elements in poetry are placed in the natural environment of the poet at that time, such as a tree or a building, which can reflect this dramatic color, so it can be seen that the drama of poetry is also influenced by the natural environment.

Tan Xusheng said, “The ‘pause' in many excellent plays is full of drama; it is precisely because this static moment contains the rich and complex psychological content of the characters, which is even better than letting the characters use lengthy lines. The lines reveal the secret of the heart, which has a greater artistic effect. The author of the quatrain also constitutes a fertile poetic environment by depicting the “still action” in similar dramas. The dramatic situation of “silence” or “pause” can inspire readers' aesthetic imagination and obtain “greater artistic effect,” for example, Li Bai's “The Resentment of the Jade Order”: “The jade order produces white dew and the long night invades Luosock. But under the crystal curtain, exquisitely looking at the autumn moon.” The whole poem only depicts the two “still movements” of the lyrical protagonists, “Empty Courtyard Long Li” and “Looking at the Moon over the Curtain.” There is not a single word of “grievance” in the poem, but the “grievance” of the characters is revealed on the back of the paper. Therefore, such an effect is produced because the poet is good at using “static movements” to construct a dramatic and nurturing poetic environment. The lyrical protagonist who stands silently in the empty courtyard is just like an actor who “pauses” in a performance on the stage. “Pause” is not Stop, it aroused the audience's doubts and expectations and mobilized the enthusiasm of the audience to play their imagination, so the readers' aesthetic imagination unfolded as promised. On the one hand, we are an audience, watching a performance of a fateful situation in front of our eyes; herself, play her and enter her situation, and feel the resentment of this jade order from her point of view. There are many such works in Tang Dynasty quatrains, such as Zhang Zhongsu's “Spring Girl,” Zhu Jiang's “Spring Girl,” Han's “Han Gong Song,” and Bai Juyi's “The Girl.” “Cage” or “stop the needle,” or “lean on” or “lean,” all of them are like actors who “pause” for a moment on the stage. Although they are silent, they can arouse the readers' corresponding aesthetic emotions, so as to obtain “bigger” artistic effect.”

The article "A Preliminary Study on the Dramatic Factors of Ancient Chinese Poetry under the Changing Geographical Environment" was retracted in 2023. Reasons: signs of a paper mill; suspected computer-generated content; unreliable results or conclusions; concerns about the data.

In ancient Chinese opera literature, we can also see such a dramatic situation of “silence.” In Wang Shifu's “The Story of the West Chamber,” when he heard that the old woman wanted Yingying to be “commensurate with her brother and sister,” Zhang Sheng was “tired and paralyzed to make a stack” and just drank it mechanically. The wine that the matchmaker handed over. In this dramatic situation, the conflict between the old lady and Zhang Sheng and others reached a climax, but the playwright arranged a “silent” action for Zhang Sheng. Obviously, the “silence” at this time implies the character's hope. The complex psychology of the peak falling to the bottom of the disappointment is worth a thousand words and more artistic than a burst of crying and hysteria. Moreover, after Wen Yingying left, Zhang Sheng made a necessary preparation for the questioning of the old lady.

### 3.2. Dramatic Plots in Tang Dynasty Quatrains

Compared with the concentrated dramatic situation, some Tang Dynasty quatrains show a time process or a certain spatial transformation, which is equivalent to a fragment of a plot. These dramatic plots contain certain dramatic conflicts and sometimes use some dramatic techniques to enhance the drama, and some of these dramatic plots even directly become the material of later dramas. Similarly, the dramatic material in poetry also contains many specific objects in natural environments, such as mountain peaks and clouds, which can constitute the dramatic material.

The article "A Preliminary Study on the Dramatic Factors of Ancient Chinese Poetry under the Changing Geographical Environment" was retracted in 2023. Reasons: signs of a paper mill; suspected computer-generated content; unreliable results or conclusions; concerns about the data.

The fundamental difference between dramatic plots and ordinary story plots is that they can constitute conflict. In the quatrains of the Tang Dynasty, this kind of dramatic conflict is mostly manifested as the inner conflict of the characters, for example, Han's “Occasionally Seen”: “To beat the sleepy and untie the skirt, and point to a statue. Seeing guests come and laugh away, rub plums in the middle of the door.” A series of actions constitute the plot, and the characters are ready to emerge: “This is exactly what the actions and expressions of a 13- or 14-year-old ancient girl who is not too shy yet, but already knows she should be shy.” It was this girl's inner conflict —wanting to see a visitor but being embarrassed to meet a visitor— that constituted the dramatic conflict.

In order to enhance the drama of the plot, this kind of Tang Dynasty quatrains also use some dramatic techniques, such as suspense and sudden turn, as shown in Figure 4. Tan Xusheng said, “Suspense is an important issue related to drama.”

The following selected Wang Jian's “Palace Ci” successfully uses the suspense technique. “Palace people clapped their hands and laughed at each other, sweeping the floor before they didn't know the steps. Begging and money arguing for borrowing, and it seems like there is no place outside?” A series of actions of the characters in the poem constitute the plot. The scene at the beginning was suspenseful: a group of court ladies laughed, shouted and clapped their hands, what made them so happy? The second sentence pointed out that the reason for the cheers was actually seeing a new unfamiliar sweeper in front of the palace steps. What is there to be happy about? The suspense at the beginning was not resolved but deepened and then the group of court ladies rushed to give money and sweep the floor, just to ask him something. What are the words so important, worthy of this group of palace maids? The suspense reached its peak. Finally, the suspense is lifted with the character's sentence: “It seems that there is nothing here outside?” While releasing the suspense, the readers also feel their inner distress and sadness behind the cheering of the characters. Because the sweeper had just entered the palace, he was so happy to be able to ask him about the scene outside the palace. It can be seen how many years they have been in the palace and how many years they have been isolated from inside and outside. The conflict between people and the environment constitutes a tragic plot, and the use of suspense techniques strengthens the tragic plot.

The article "A Preliminary Study on the Dramatic Factors of Ancient Chinese Poetry under the Changing Geographical Environment" was retracted in 2023. Reasons: signs of a paper mill; suspected computer-generated content; unreliable results or conclusions; concerns about the data.

The dramatic plot pieces of some quatrains even provide the plot directly for the play, for example, in Du Mu's “Quanjue Passing Huaqing Palace”: “Looking back at Chang'an, there are piles of embroidered embroidery, and thousands of gates on the top of the mountain are opened one after another. When a concubine of Hongchen laughs, no one knows that it is a lychee.” “Incoming Fruit” reappeared in the first out. He took advantage of the style of drama and transformed the plot into a series of dramatic scenes and more tortuous storylines: the envoys from Nanhai and Shuzhou rushed all the way to get fresh lychees to the court as soon as possible and were killed. The old man selling divination trampled the peasants' crops. The two are still vying for good horses at the poststation. Another example is Cui Hu's quatrain “Tiducheng Nanzhuang,” which was cited by the Ming Dynasty dramatist Meng Chengshun as plot material. In the novel, the peach blossoms on the human face are red with each other. Where will the human face go now? The peach blossoms are still smiling in the spring breeze,” so the twists and turns of the plot are full of poetic and picturesque. The same is true of Leng Chaoyang's quatrain “Send the Red Thread,” which directly became the material for the work “Red Thread Girl” by Liang Chenyu, a playwright in the Ming Dynasty. The abovementioned drama writers keenly captured the dramatic elements in these widely read Tang quatrains, used them directly as drama materials, and greatly developed the drama in them. The element of peach blossom is used in the ancient poems, and the peach blossom represents the natural environment, so the natural environment influences the literary color of the poetry by influencing the poet's creative inspiration.

## 4. Dramatic Discourses in Tang Dynasty Quatrains

There are also some Tang Dynasty quatrains that neither express the concentrated situation nor show certain plot fragments. The whole text seems to be the author's endorsement of the characters speaking to a specific object. Narrative discourse is different, but has the characteristics of dramatic discourse.

Most of the lyrics used for music in the Tang Dynasty were excellent five-seven-character quatrains. Tang quatrains, which can sing and can be enjoyed by both the refined and the popular, are close to dramatic discourse in their clear and subtle features. In some lyrical Tang Dynasty quatrains, the poet puts himself in the shoes of the characters he endorses and the characters' language is full of personality, which is similar to the personality of the language of the characters in the drama of the endorsement style. The drama wheel of the Tang Dynasty is shown in Figure 5. The main reason why these Tang Dynasty quatrains can be regarded as dramatic discourses is that the objects of the characters' dialogues or monologues are specific objects determined by the characters themselves in a specific situation and belong to the readers and listeners in the works, not outside the works. This is the biggest difference between dramatic discourse, lyrical discourse, and narrative discourse, the latter two being aimed at readers and listeners outside the works. At the same time, these discourses are all words that characters must say in a specific time, place, and environment, for their own purposes, to take action to a specific object, so they have a certain action.

The article "A Preliminary Study on the Dramatic Factors of Ancient Chinese Poetry under the Changing Geographical Environment" was retracted in 2023. Reasons: signs of a paper mill; suspected computer-generated content; unreliable results or conclusions; concerns about the data.

First of all, the clear and implicit language features of these Tang quatrains are similar to the dramatic discourse.

Such excellent Tang Dynasty quatrains are often sung with music, so that all the listeners can understand them, so the language should be clear and clean, but also to make the listeners emotional, the content should be profound and tortuous. Therefore, it corresponds to the clear and implicit characteristics of dramatic discourse, for example, Shen Xun's “Feast of Poems”: “Don't hit the wild goose from the south, fly from him to the north. When you hit a double hit, don't send the two to separate.” The lyrical protagonist is pitiful and sympathetic, and the complex mentality of empathy is also understood by the listeners.

Second, the characters in this kind of Tang Dynasty quatrains have distinct personalities, similar to the characteristics of dramatic discourse.

In addition to being clear and subtle, dramatic discourse must also be able to express the personality of the characters, as Li Yu, a drama theorist in the Qing Dynasty, said, “Make sure your heart is subtle and spit out casually. Make it superficial.” That is to say, the characters' language must be able to show the little-known and difficult-to-understand secrets in the characters' hearts, and this display must be “spit out,” that is, naturally and clearly. It is also necessary to “say one person, and Xiao one person,” that is, the words are like the person and the character's character can be seen from the language of the character. In the quatrains of the Tang Dynasty, we can see some lyrical quatrains, imitating the tone of the characters they represent. Even the same women have different personalities.  Table 3 lists the distinctive characters in the four lines of the Tang Dynasty.

The article "A Preliminary Study on the Dramatic Factors of Ancient Chinese Poetry under the Changing Geographical Environment" was retracted in 2023. Reasons: signs of a paper mill; suspected computer-generated content; unreliable results or conclusions; concerns about the data.

Third, the lyrical protagonists in this kind of Tang Dynasty quatrains have definite speaking objects in the works.

Both characters speak by themselves, and the lyrical discourse is aimed at readers or listeners outside the system of the work, while the lyrical protagonists of this type of Tang Dynasty quatrains speak from the internal system of the work, so they are not lyrical discourse and have the characteristics of dramatic discourse. For example, in Shen Xun's “Feasting Poems,” the lyrical protagonist speaks to the man in front of the wild goose who he (she) wants to dissuade. The outspoken swordsman in Jia Dao's “The Swordsman” speaks to his confidant who is worthy of a sword. The lyrical protagonists in Li Bai's “Ba Nuci,” Meng Jiao's “Ancient Resentment,” and Zhang Jiuling's “From Your Majesty Has Come” are all their “Langjun,” the difference is only that some are in front of you and some are not in front of you.

Finally, the discourse of this kind of Tang Dynasty quatrain also has the characteristics of action similar to the dramatic discourse.

Most of the words spoken by the lyrical protagonist of this kind of Tang quatrains are what he or she must say at a specific time, place, and environment, for his or her own purpose, to take action against a specific object. Therefore, it has the characteristics similar to the action of dramatic discourse. Typical examples in this regard are the first two poems of Cui Hao's “Changgan Song,” the two poems are like questions and answers for children on the river. First, the woman asked, “Where does Jun's house live?” Without waiting for the other party's answer, she said, “The concubine lives in Hengtang.” It's a fellow countryman.” In a series of words, the image of a girl who is both enthusiastic and measured, both hearty and reserved, suddenly appeared on the paper. Behind the simple language of the characters, we can imagine a series of actions of the characters: the girl fell in love with the young man among the countless boats that came and went and tried her best to make her boat catch up with the young man's boat. The second song is the answer for the young man: “My home is near the water of Jiujiang River, and I come and go to the side of Jiujiang River. We are both from Changgan, but we didn't know each other when we were young.” Behind the simple language of the character, we can feel his inner actions: the joy of meeting the villagers and a trace of regret for seeing each other late. This is also the emotional reaction that the girl's words caused in his heart. The dialogue between the two characters seems simple, but they are actually full of action and subtext. The characters are divinely shaped, and even the atmosphere of the scene is in front of us, as if the poet used forty words to show” us a love drama, just as Zhu Guangqian said, “It's like a scene …. The moment taken from the life and life of the artist …. This is a moment, art infuses it with life, and it becomes eternal … .”

The article "A Preliminary Study on the Dramatic Factors of Ancient Chinese Poetry under the Changing Geographical Environment" was retracted in 2023. Reasons: signs of a paper mill; suspected computer-generated content; unreliable results or conclusions; concerns about the data.

To sum up, compared with the drama in the drama literature, due to the influence of the natural geographical environment, the plot of the four lines in the Tang Dynasty is not complicated, often just fragments, the conflict is not fierce, the relationship between the characters is not complicated, and the movements of the characters are very simple. However, it has been recited by the population for a long time. It can sing and be appreciated by both the refined and the popular. It is loved by all social classes and has many similarities with ancient Chinese opera. It goes without saying that Chinese drama literature draws nourishment from Chinese poetry in many ways, but the dramatic factor in the quatrains of the Tang Dynasty, which has been recited by the population for thousands of years and has a wide and lasting power of dissemination, should be one of the most influential factors in Chinese drama literature. It is an aspect that cannot be ignored and thus gets due attention and research.

## 5. Conclusion

This paper studies the cultural characteristics of different historical background and the specific influence of natural geographical environment on the traditional culture, explores the drama factors in the four lines in the Tang Dynasty, and determines the dramatic elements in the Tang Dynasty poetry. The geographical study of ancient Chinese poetry drama factors has certain significance.

In a word, poetry and literature, as an important human spiritual activity content and the way of life existence, will undoubtedly be affected by the geographical environment. Therefore, when studying literary works, we should not only pay attention to the author's life experience and time background but also pay attention to the influence of geographical environment in the process of literary work creation, which is more conducive to our comprehensive understanding and appreciation of literary works.

## Figures and Tables

**Figure 1:** Natural geographical environment.

**Figure 2:** Forms of ancient civilizations in the world.

**Figure 3:** Dramatic factors in Tang Dynasty quatrains.

**Figure 4:** Dramatic techniques used in Tang Dynasty quatrains.

**Figure 5:** Dramatic discourses in Tang Dynasty quatrains.

The article "A Preliminary Study on the Dramatic Factors of Ancient Chinese Poetry under the Changing Geographical Environment" was retracted in 2023. Reasons: signs of a paper mill; suspected computer-generated content; unreliable results or conclusions; concerns about the data.

**Table 1:** Differences in culture between north and south caused by changes in geographical environment.

The cultural consistency of the north is relatively strong	The southern cultures have their own characteristics
In the central and northern regions of China, poetry represented by the “Book of Songs” appeared. It is characterized by elegance and gentleness, in line with etiquette, and with realism as the main feature	In the south, poems such as “Li Sao” appear, which are very different from the Book of Songs, showing a blurred and magical romantic color

**Table 2:** Dramatic situations in Tang Dynasty quatrains.

Meng Jiao “Farewell to the ancients”	If you want to leave Lang Yi, where is Lang now? Don't hate returning late, do not go to Linqiong	The characters are the lyrical protagonist and the “Lang,” the location is the two people's homes, the time is the moment of “wanting to say goodbye,” the events are parting words, and the contradictions and conflicts are concentrated in the inner conflict of the lyrical protagonist. Secondly, this moment is mostly the moment before the conflict comes.

Wang Jian “Palace Ci”	The old courtyard was unbearable to repair, and the recent edict Xuanhui put up the building. Hearing that there is a new beauty entering, there is no sorrow in the sixth palace	What the poet chooses is the moment before the conflict between the “beautiful woman” who has not yet entered and the “six palace” concubines and concubines. Again, this particular moment includes pre-pregnancy and post-conception. It contains and implies “many line events” before and after this moment.

Kim Chang-Seo “Spring resentment”	When the yellow yinger is played, do not teach the branch to cry. When I cried, I was shocked and dreamed of a concubine, and I could not get west of Liaoning	The poet appropriately selects the moment when the young woman in her boudoir “plays a warbler and seeks a dream” before going to bed. From this moment, readers can infer that the lyrical protagonist must be separated from her husband who joined the army. There is no news for a long time, and longing and worry coexist. However, a weak girl in her boudoir has no other way to find other than to ask for a dream. The dream is so urgent, so she has a conflict with the “Huang Ying” who may have a startling dream. In order not to be disturbed by such a dream “Fighting warblers.” But after “playing the warbler,” will you be able to fall asleep and dream? Even if you dream, will you be able to dream of the husband who is in the army? This moment before and after pregnancy can prompt readers to develop rich associations.

**Table 3:** Characters with distinct personalities in Tang Dynasty quatrains.

Chao Cai “Midnight song”	“Nong has cut the cloud, and Lang has also divided his hair. Looking for no one, wan makes a concentric knot” “Jade fingers on the bright window, nails are like crystal. Cut Tejiro, talk and go hand in hand”	What we see is a happy girl who is in love

Li Yi “Jiangnan song”	“Marry Qutang Jia, and the court missed the concubine period. If I knew that the tide has faith, marry and follow the tide”	We clearly saw a businesswoman in her boudoir who was extremely resentful

The article "A Preliminary Study on the Dramatic Factors of Ancient Chinese Poetry under the Changing Geographical Environment" was retracted in 2023. Reasons: signs of a paper mill; suspected computer-generated content; unreliable results or conclusions; concerns about the data.

## Data Availability

The labeled dataset used to support the findings of this study is available from the author upon request.
